# Role of Acute Physiology, Age, and Chronic Health Evaluation (APACHE) II Score in Predicting Outcomes of Peritonitis Due to Hollow Viscous Perforation: A Prospective Observational Study

**DOI:** 10.7759/cureus.20155

**Published:** 2021-12-04

**Authors:** Seshu Kumar Bylapudi, Sugunesh Nanjan, Sadhasivam Ramasamy, Amudhan Kannan, Ketan Kantamaneni, Shalini Nangireddi, Lakshmi Malvika Atluri, Suresh Kondi, K S Rajkumar

**Affiliations:** 1 General Surgery, Pilgrim Hospital, Boston, GBR; 2 Surgery, Royal Gwent Hospital, Newport, GBR; 3 General Surgery, Milton Keynes University Hospital, Milton Keynes, GBR; 4 Surgery, Jawaharlal Institute of Postgraduate Medical Education and Research, Puducherry, IND; 5 Surgery, Dr. Pinnamaneni Siddhartha Institute of Medical Sciences and Research Foundation, Gannavaram, IND; 6 Obstetrics and Gynaecology, Lourde Hospital, Kannur, IND; 7 Surgery, Dr. Pinnamaneni Siddhartha Institute of Medical Science, Gannavaram, IND; 8 Surgery, Citi Neuro Centre, Hyderabad, IND; 9 General Surgery, Kovai Medical Center, Coimbatore, IND

**Keywords:** mortality, morbidity, surgery, prognosis, peptic ulcer disease, apache, score, peritonitis, perforation, outcome

## Abstract

Background

The Acute Physiology and Chronic Health Evaluation II (APACHE II) is the most commonly used severity-of-disease scoring system in ICUs worldwide. There is a paucity of data describing the role of APACHE II score in predicting outcomes of peritonitis due to hollow viscous perforation. This study aims at identifying the importance of the APACHE II score in predicting outcomes of patients with peritonitis secondary to hollow viscus perforation.

Methods

The study is a prospective, observational study that included all the patients diagnosed with perforation peritonitis who underwent emergency laparotomy and were admitted to the Department of Surgery from May 2017 to May 2018. APACHE II scores were assigned to all patients in order to calculate their individual risk of mortality before undergoing emergency surgery. The accuracy in outcome prediction of the APACHE II system was assessed by means of receiver operating characteristic (ROC) curve and Pearson correlation coefficient and its significance test.

Result

A total of 50 patients with perforation peritonitis were included in this study. Peptic ulcer disease was the major etiology leading to perforation in 54% of patients, followed by gangrenous bowel. The mean APACHE II score was 9.54. Out of the 50 patients, seven patients succumbed to the illness. All the seven patients whose APACHE II score > 16 developed systemic complications, and three of them developed a local complication.

Conclusion

APACHE II score correlated well with the outcome in the current study, and APACHE II score also correlated well with the hospital and ICU stay.

## Introduction

One of the most widely used scoring systems for assessing the severity of disease in ICUs is the Acute Physiology and Chronic Health Evaluation II (APACHE II). Within the first 24 hours of patient admittance, the worst value for each physiological variable is calculated into an integer score from 0 to 71. Higher APACHE II scores correlate to the severity of the disease and a higher hospital mortality risk. Knaus et al. presented the first APACHE model in the 1980s [1].

Peritonitis is the inflammation of the peritoneum. It is most commonly due to localized or generalized infection caused by various probable factors. Based on the nature and source of microbial contamination, peritonitis is divided into three stages, viz., primary, secondary, and tertiary peritonitis. Primary peritonitis is the infection of the peritoneum without any visceral perforation and is usually from an extraperitoneal source. It is monomicrobial in origin. Secondary peritonitis is the most common, and it is due to the perforation of the viscera. It is from an intraperitoneal source. Examples include duodenal ulcer perforation, infectious like typhoid, blunt trauma of abdomen, etc.

If left untreated or treatment fails, peritonitis usually develops into a fatal tertiary stage. Although advances are available in diagnosis, surgical techniques, antimicrobial therapy, and intensive care support, the morbidity and mortality associated with this are high [2]. Superimposed infections can lead to bacterial contamination of the peritoneal cavity, ultimately progressing to abscess formation and sepsis, which is associated with a high mortality rate. Patients often present with symptoms such as abdominal pain or distention, fever, and tachycardia. Studies in the literature have reported that the factors associated with high morbidity and mortality in patients with peritonitis are malnutrition and intake of immunosuppressive agents. Therefore, it is crucial to recognize and treat sepsis early to improve patient outcomes. Surgical intervention is often required to control the septic focus, but individualized treatment comparing the risks and benefits of surgery to more conservative management must be considered [3].

Despite recent advances in surgical techniques and intensive perioperative care, mortality rates remain high. Thus, it is important to predict the postoperative outcome by conducting preoperative examinations and evaluating the patient’s condition [4]. Severity scoring is a valuable tool for assessing and quantification of the severity of acute illness. Currently, Acute Physiological and Chronic Health Evaluation (APACHE II) scoring system is the best available method for risk stratification in abdominal sepsis [5].

However, there is scanty literature describing the role of APACHE II score in predicting outcomes of peritonitis due to hollow viscous perforation. This study aims at identifying the importance of the APACHE II score in predicting outcomes of patients with peritonitis secondary to hollow viscus perforation.

## Materials and methods

The study is a prospective, observational study that was conducted in tertiary-care hospital Kovai Medical Centre and Hospital, Coimbatore, India. Institutes ethics committee approval was obtained for conducting this study (KMC/IEC/208503).

Eligibility criteria

We included all the patients diagnosed with perforation peritonitis who underwent emergency laparotomy and were admitted to the Department of Surgery and observed in the surgical intensive care unit (SICU) from May 2017 to May 2018. We excluded the patients who had blunt trauma to the abdomen and associated solid organ injury, vascular injury, neurological injury, or fracture.

Diagnosis of peritonitis

A diagnosis of peritonitis due to hollow viscus perforation was made by history and clinical examination, radiologically by evidencing the presence of air under the diaphragm and later confirmed during the exploration laparotomy.

We assigned APACHE II scores to all patients before undergoing surgery in order to calculate their individual risk of mortality. We used the receiver operating characteristic (ROC) curve, Pearson correlation coefficient, and its significance test to estimate the accuracy in outcome prediction of the APACHE II system.

Patients included in this study had various etiologies causing perforation, such as peptic ulcer disease (PUD), typhoid, blunt injury abdomen, and malignancy.

We calculated the APACHE II scores using the method of the Knaus et al. study [6]. A comparison of the observed death rate to the predicted death rate for the study group was made as a part of the analysis.

Statistical analysis

All the data were entered into the SPSS spreadsheet, and the analysis was done in SPSS version 20.0 (SPSS Inc., Chicago, IL, USA). All the statistical tests were examined with a 5% ( p-value ≤ 0.05) level of significance. An unpaired t-test was used to compare the mean and standard deviations of two independent variables.

The accuracy of outcome prediction by the APACHE II system was assessed by using the ROC curve and Pearson correlation test.

## Results

A total of 50 patients with perforation peritonitis were included in this study. The mean age of the study population was 43.68 years. Of the 50 patients, 42% of patients fell into the 31-50 years age group, and 36% of patients fell into the 51-70 years age group. Out of the 50 patients, 78% of patients were males, and the remaining were females.

Of the etiological factors leading to perforation, Peptic ulcer disease forms the major etiology leading to perforation in 27% of patients, followed by gangrenous bowel in 14% of patients. The etiological distribution of the patients diagnosed with peritonitis is shown in Table 1.

**Table 1:** Etiology of peritonitis

Diagnosis	N (%)
Peptic ulcer disease	27 (54)
Appendicular perforation	5 (10)
Blunt trauma abdomen	5 (10)
Postmedical-termination of pregnancy	1 (2)
Malignant sigmoid colon perforation	1 (2)
Gangrenous bowel	7 (14)
Tuberculous peritonitis	2 (4)
Typhoid	2 (4)

Postoperative complications

A total of 16 patients developed postoperative local complications. The most common postoperative complication was surgical site infection (SSI). A total of 19 patients developed systemic complications following surgery, of which sepsis and acute respiratory distress syndrome (ARDS) were the leading complications. Table 2 shows the incidence of postoperative local and systematic complications in our study population.

**Table 2:** Incidence of postoperative complications

Complication:	N (%)
Local Complications:	
Anastomotic leak	1(2)
Fecal peritonitis	4(8)
Intra-abdominal abscess	2(4)
Surgical site infection	9(18)
Systemic complications:	
Acute respiratory distress syndrome	7(14)
Acute renal failure	1(2)
Congestive cardiac failure	2(4)
Sepsis	9(18)

On analyzing the APACHE II score of the patients, the mean APACHE II score was 9.54. Of the total patients, 24% were in the APACHE II score 11-16 category, 34% were in the APACHE II score 6-10 category, and 28% of the patients were in the APACHE II score 0-5 category. Out of the 50 patients, seven patients succumbed to the illness.

All the seven patients whose APACHE II score > 16 developed systemic complications, and three of them developed a local complication. Out of 14 patients having APACHE II scores (0-5), only two patients developed local complications. And all patients survived.

Hospital and ICU stay

On analyzing the hospital and ICU stay, the mean hospital stay was 9.79 days, and the mean ICU stay was 0.64 days in patients with the APACHE II score of 0-5. In patients with APACHE II scores of 6-10, the mean hospital stay was 11.29 days, and the mean ICU stay was 0.82 days. In patients with APACHE II score 11-16, the mean hospital stay was the longest, and it was 12.42 days, and the mean ICU stay was 1.08 days.

Mortality

Table 3 shows 100% mortality was in APACHE II score > 20. There was no mortality in the APACHE II score (0-5). It also shows the comparison of various parameters in APACHE score categories.

**Table 3:** Comparison of various parameters in various APACHE II score categories

APACHE II scores	0-5	6-10	11-15	16-20	>20
Local complications [N (%)]	2 (14.2)	6 (35.2)	5 (41.6)	1 (25)	2 (66.6)
Systematic complications [N (%)]	2 (14.2)	5 (29.4)	5 (41.6)	4 (100)	3 (100)
Duration of stay (mean ± SD)	9.79 ± 5	11.29 ± 3.42	12.42 ± 4.94	4.00 ± 1.83	6.33 ± 3.79
Duration of ICU stay (mean ± SD)	0.64 ± 0.84	0.82 ± 0.64	1.08 ± 0.79	2.25 ± 0.50	1.67 ± 0.58
Mortality [N (%)]	0 (0)	0 (0)	1 (8)	3 (75)	3 (100)

Comparison of survivors and non-survivors

The mean age in survivors was 41.58 years, and in non-survivors was 56.57 years, and it did not show any significant difference between the two groups.

The mean hospital stay in survivors was 11.02 days, and in non-survivors was 5.57 days, and it showed a significant difference between the two groups. Like the mean hospital stay, the mean ICU stay also showed a statistically significant difference between the two groups.

The mean APACHE II score (7.93 vs. 19.43 in survivors vs. non-survivors) also showed a significant difference between the two groups.

Table 4 shows the comparison between survivors and non-survivors in various parameters.

**Table 4:** Comparison of parameters between the survivors and the non-survivors

Parameters	Survivors	Non-survivors	P-value
Age (mean ± SD)	41.58 ± 15.27	56.57 ± 10.1	0.016
No. of Stay (mean ± SD)	11.02 ± 4.5	5.57 ± 3.41	0.004
ICU Days (mean ± SD)	0.84 ± 0.75	2.00 ± 0.58	< 0.001
Score (mean ± SD)	7.93 ± 3.91	19.43 ± 3.10	< 0.001

## Discussion

The primary objective of this study was to assess the outcomes of patients having perforation peritonitis using the APACHE II score.

In the current study, the mean age was 43.68 ± 15.49 years, which is comparable to 40.4 years in the study done by Kitara et al. [7]. The incidence among males was more than the females in the ratio of 3.2:1. Huttunen et al., in their study, also reported male preponderance in cases with perforation peritonitis [8].

Cause of perforation

In our study, the most common cause of perforation peritonitis was PUD, which was seen in 54% of the patients. PUD most commonly arises from the ulcers of the first part of the duodenum [9-11]. In our study, the second most common cause of perforation peritonitis was appendicular perforation peritonitis, whereas, in studies by Afridi et al. and Khan et al., tubercular perforation peritonitis reported the incidence to be 21% and 22%, respectively [9,11].

Post-op complications

In our study, we identified that the postoperative complications were significantly higher in the patient having an APACHE II score of more than 10 at the time of admission. The most common complication was SSI and was seen in 18% of the cases. SSI represents one of the most important complications occurring postoperatively following surgical procedures, and the SSI incidence is higher following gastrointestinal surgeries compared to any other surgery [12]. It contributes to the majority of morbidity and mortality in patients undergoing GI surgeries.

Analysis showed 19 patients developed systemic complications. Sepsis and ARDS were the leading complications accounting for 9% and 7%, respectively. As the APACHE II score includes chronic health evaluation into account, susceptible patients with higher scores can be sensed earlier and appropriately monitored for deterioration.

APACHE score and hospital and ICU stay in survivors vs non-survivors

The mean hospital stay and the mean ICU stay in survivors also showed a significant difference. In Bohnen et al. study, the mean duration of hospital stay following treatment in survivors was 11.02 days as compared to 18 days [13].

APACHE score and outcome

In this study, 31 patients belonged to the low-risk category with an APACHE score of 0-10, and 16 patients belonged to the medium-risk group with an APACHE score of 10-20, and three patients were in the high-risk group of APACHE score > 20. Out of these patients, the high-risk group had a 100% mortality rate, whereas 100% of patients in the low-risk group and 75 % of patients in the medium-risk group were discharged in a satisfactory manner.

Analyzing outcomes in terms of complication, we identified that out of seven patients having APACHE II score > 16, all develop systemic complications, and three patients develop a local complication. Out of 14 patients having APACHE II score (0-5), only two patients developed a local complication, and all patients survived.

In studies conducted by Bohnen et al. and Adesunkanmi et al., the mean APACHE score among survivors was 8 (low-risk group) and among non-survivors was 22.4 (high-risk group). These studies concluded that mortality is directly linked with higher APACHE II scores [13,14].

Using ROC analysis, the area under the curve was found to be 99.5%. The correlation of APACHE-II score and predicted death rate showed perfect correlation, with r = 0.729. Kulkarni et al. analyzed the APACHE II score in peritonitis and achieved an area under the curve using ROC to be 98.4%. Our study produced a better result compared to Kulkarni et al. [15]. The APACHE-II system was found to be accurate in group outcome prediction as assessed by the ROC curve and Pearson correlation coefficient and its significance test. This value is higher when compared to values found by other workers who evaluated the APACHE-II scoring system in ICU patients, including both surgical and medical patients in their study group.

The APACHE-II scoring system can be used to assess group outcomes in patients with peritonitis due to hollow viscous perforation. However, it did not provide sufficient confidence for outcome prediction in individual patients.

Our study has a few limitations. This study is a single-center, and this does not represent the whole population. A multicenter study is needed to make a better prediction of the outcome. Surgical intervention contributes mainly to the outcome of these patients. Modality and strategies of surgical management were not studied. The study population was less when compared with similar studies done by others because of time constraints. We want to continue this study further to gain a good sample size for statistical analysis. Single etiology for perforation was not taken into account owing to less volume. Taking up a single cause will help in better statistical analysis for predicting outcomes.

## Conclusions

We can conclude from the study that the APACHE II score can be used to predict the outcome of patients who presents with hollow viscus perforation. Patients with an APACHE II score of more than 20 have a very high risk of mortality postoperatively and those who have a score of more than 15 are at risk of developing systemic complications. In addition, the APACHE II score can also correlate with the hospital and ICU stay. We recommend future studies with a large sample size be conducted to report results with much higher clarity.
